The article "Outer Membrane Protein A (OmpA) of Shigella flexneri 2a Induces TLR2-Mediated Activation of B Cells: Involvement of Protein Tyrosine Kinase, ERK and NF-κB" was retracted in 2020. Reasons: original data or images not available; concerns about the data; concerns about the images; concerns about the results or conclusions.

# Outer Membrane Protein A (OmpA) of *Shigella flexneri* 2a Induces TLR2-Mediated Activation of B Cells: Involvement of Protein Tyrosine Kinase, ERK and NF-κB

**DOI:** 10.1371/journal.pone.0109107

**Published:** 2014-10-06

**Authors:** Rajsekhar Bhowmick, Debasis Pore, Manoj K. Chakrabarti

**Affiliations:** Division of Pathophysiology, National Institute of Cholera and Enteric Diseases, Kolkata, West Bengal, India; Queen's University Belfast, United Kingdom

## Abstract

B cells are critically important in combating bacterial infections and their differentiation into plasma cells and memory cells aids bacterial clearance and long-lasting immunity conferred by essentially all vaccines. Outer membrane protein A (OmpA) of *Shigella flexneri* 2a has been demonstrated to induce the production of IgG and IgA *in vivo* following immunization of mice through intranasal route, but the direct involvement of B cells in OmpA-mediated immune regulation was not determined. Consequently, we investigated whether OmpA can modulate B cell functions and identified the molecular events involved in OmpA-induced B cell immune response *in vitro*. We show that OmpA of *S. flexneri* 2a activates B cells to produce protective cytokines, IL-6 and IL-10 as well as facilitates their differentiation into antibody secreting cells (ASCs). The immunostimulatory properties of OmpA are attributed to the increased surface expression of MHCII and CD86 on B cells. We also report here that B cell activation by OmpA is mediated strictly through recognition by TLR2, resulting in initiation of cascades of signal transduction events, involving increased phosphorylation of protein tyrosine kinases (PTKs), ERK and IκBα, leading to nuclear translocation of NF-κB. Importantly, a TLR2 antibody diminishes OmpA-induced upregulation of MHCII and CD86 on B cell surface as well as significantly inhibits B cell differentiation and cytokine secretion. Furthermore, we illustrate that B cell differentiation into ASCs and induction of cytokine secretion by OmpA are dependent on PTKs activity. Moreover, we identify that OmpA-induced B cell differentiation is entirely dependent on ERK pathway, whereas both NF-κB and ERK are essential for cytokine secretion by B cells. Overall, our data demonstrate that OmpA of *S. flexneri* 2a amplifies TLR signaling in B cells and triggers B cell immune response, which is critical for the development of an effective adaptive immunity to an optimal vaccine antigen.

## Introduction

Shigellosis, a leading cause of human diarrhoeal disease, remains an imperative cause of childhood morbidity and mortality in the developing countries [1]. Globally 164 million cases of shigellosis occur annually, with over 1.1 million cases resulting in death per year [1]. The worldwide prevalence of *Shigella* species resistant to antimicrobial drugs [2] creates the development of an effective vaccine more pressing. Despite advancement in *Shigella* vaccine research, no approved vaccine is currently available to rheostat shigellosis.

The use of bacterial outer membrane proteins as vaccine candidates has been emphasized in the recent years [3]–[5]. We have previously explored that outer membrane protein A (OmpA) of *Shigella flexneri* 2a possesses the essential characteristics of a potential vaccine antigen, which includes crossreactivity, surface exposed epitope and conservation among strains [6], [7]. The mechanism of immunogenicity of *S. flexneri* 2a OmpA as vaccine antigen correlates with its ability to activate macrophages with the surface expression of MHCII, CD80 and CD40 [8], which in turn, facilitates stimulation of adaptive immune response by activation of CD4^+^ T cells [9]. TLR2 has been recognized as an indispensible factor in OmpA-mediated coordination between the innate and adaptive arms of the immune response [9]. Moreover, OmpA evokes strong protective immune response against the homologous virulent strain in mice without addition of exogenous adjuvants [10] and that the immunity might involve synergy among the cellular and humoral immune responses. Intranasal immunization of mice with OmpA induces antigen specific IgG and IgA production in both the systemic and mucosal compartments [10], demonstrating participation of B cells in OmpA-induced protective immune response *in vivo*. However, the effect of *S. flexneri* 2a OmpA on B cells has not been delineated yet. Hence, the present study has been instigated to illuminate whether OmpA can directly activate B cells and identify the molecular mechanism behind it.

B cells play a fundamental role in humoral immunity by producing high-affinity antibodies for immunological protection against pathogens [11], [12] and regulate CD4^+^ T-cell responses to foreign antigens [13], function as antigen-presenting cells [14], produce cytokines [15], provide co-stimulatory signals [16], and promote naïve CD4^+^ T-cell differentiation into T-helper 1 or 2 subsets [17]. B cell receptor (BCR) signaling plays pivotal role in the generation and activation of B- lymphocytes [18]. Besides BCR, recent studies reveal that B cells are directly informed about the presence and nature of pathogens by sensing microbial conserved structures, termed pathogen-associated molecular patterns (PAMPs) by the pattern recognition receptors, such as Toll like receptors (TLRs), expressed on there surface [19], [20]. Engagement of TLRs by microbial products results in homodimerization and recruitment of the adaptor molecule MyD88 leading to activation of various intracellular signaling pathways such as NF-κB and mitogen-activated protein (MAP) kinases that regulate secretion of cytokines [21], upregulation of costimulatory molecules B7-1 (CD80) and B7-2 (CD86) [22], resulting in B cells activation, proliferation and differentiation of naïve B cells, including immunoglobulin (Ig) class switch DNA recombination (CSR), all of which greatly influence the adaptive immune response thereby allows the host to more efficiently eradicate the invading pathogens from the body [23], [24].

In this study we reveal that OmpA of *S. flexneri* 2a stimulates and induces proliferation and differentiation of splenic B cells. The activated B cells secrete effector cytokines like IL-6 and IL-10 as well as upregulate surface expression of class II major histocompatibility complex (MHC) and costimulatory molecule CD86. The immunopotentiating ability of OmpA is dependent on TLR2 expression and activation of downstream signaling molecules, such as, ERK phosphorylation and NF-κB nuclear translocation, as demonstrated by absence of immune response by TLR2, NF-κB or ERK inhibited B cells to OmpA. Our data illustrate that OmpA is a potent activator of B cell immune response and provide further evidences that OmpA of *S. flexneri* 2a can be a potential candidate for future development of an ideal subunit vaccine against shigellosis.

## Materials and Methods

### Ethics statement

Animal care and experiments were conducted according to the guidelines established by the National Institute of Cholera and Enteric Diseases (NICED) ‘Institutional Animal Ethics Committee’ (IAEC) concerned under the guidance of the ‘Committee for the Purpose of Control and Supervision of Experiments on Animals’ (CPCSEA), Govt. of India. All animal experiments were approved by NICED ‘Institutional Animal Ethics Committee’ (approval no. 18/7-6-2000). Euthanasia of mice was done with CO_2_ inhalation followed by cervical dislocation before spleen harvesting.

### Mice

BALB/c mice were originally purchased from Jackson Laboratory (Bar Harbor, ME). All mice were maintained and bred in specific pathogen-free barrier facility at the National Institute of Cholera and Enteric Diseases (NICED), Kolkata, India and used at the age of 8 to 12 weeks.

### Cell line and transfection

The HEK293 cell line (ATCC) was cultured in Dulbecco's modified Eagle's medium (Invitrogen) supplemented with 10% fetal bovine serum and 10 µg/ml of ciprofloxacin (Sigma). The cells were grown in 5% CO_2_ at 37°C to confluent monolayers in 24-well plates (BD Falcon). HEK293 cells were plated in 6-well tissue culture plates (4×10^5^ cells/well). Using TransFast transfection reagent (Promega), the cells were transfected with pNF-κB-MetLuc2-Repoter vector (Clontech) and followed by human NOD1 or NOD2 expression plasmids (InvivoGen). OmpA (5 µg/ml) or muropeptides (diaminopimelic acid-containing muramyl tripeptide [M-triDAP] for NOD1 and muramyl dipeptide [MDP] for NOD2, both at 100 nM) were added to the cell culture medium at the time of transfection and the synergistic NF-κB-dependent luciferase activation was examined following 16 h of coincubation by using the Ready-To-Glow Secreted Luciferase Reporter Assay System (Clontech), according to the manufacturer's instructions. M-triDAP was purchased from InvivoGen and MDP was from Sigma.

### Antibodies and reagents

Phycoerythrin (PE)-conjugated anti-mouse CD19 (Clone: 1D3), FITC-conjugated anti-mouse MHC class II (I-A/I-E), FITC-conjugated anti-mouse CD80 (Clone: 16-10A1), Hamster IgG2 κ isotype control FITC, FITC-conjugated anti-mouse CD86 (Clone: GL1), Rat IgG2a κ isotype control FITC antibodies were purchased from BD Biosciences. Purified anti-mouse TLR1 (Clone: eBioTR23), Rat IgG2a κ isotype control purified, Anti-rat IgG Biotin, Streptavidin PE, FITC-conjugated anti-mouse TLR2 (Clone: 6C2), Rat IgG2b κ isotype control FITC, PE-conjugated anti-mouse TLR4 (Clone: UT41), Mouse IgG1 κ isotype control PE antibodies were obtained from eBioscience. Purified anti-mouse TLR6 (Clone: 418601) was purchased from R&D Systems. Detoxi-Gel Endotoxin Removing Columns were purchased from Pierce. Antibodies to phospho-ERK, ERK, phospho-p38, p38, phospho-JNK, JNK, phospho-IκB, Lamin B1 and α-Tubulin were obtained from Cell Signaling Technology. α-p65, IκB and β-Actin antibodies were purchased from Santa Cruz Biotechnology. Biotin-Conjugated Anti-Phosphotyrosine antibody (clone 4G10) was obtained from Millipore.

### Immunogen

OmpA of *S. flexneri 2a* was expressed in *E. coli* BL21 (DE3) and purified as described previously [10]. The protein obtained was about 95% in purity (**Figure S1**) without glycosylation. The lipopolysaccharide present (different stocks of purified OmpA samples contained 0.78 to 1.3 EU of LPS/ml) in the recombinant OmpA was removed by passing the protein through Detoxi-Gel endotoxin removing resin and S3Δ peptide affinity gel columns, respectively, that resulted in virtually pyrogen-free OmpA containing <0.0001 EU of LPS/ml. A *Limulus* amoebocyte lysate chromogenic assay with Kinetic-QCL (Lonza) was performed to determine the level of LPS present in recombinant OmpA. To exclude the possibility of peptidoglycan (which can activate cells via NOD1 and NOD2) contamination in our recombinant OmpA preparations, we used HEK293 cells transfected with NOD1 or NOD2 expression plasmids and an NF-κB-dependent luciferase reporter gene. As shown in **Figure S2**, the recombinant OmpA showed a negligible NF-κB activation, which was comparable to untreated control. As positive controls, we used M-triDAP for NOD1 and muramyl dipeptide for NOD2. These results confirm the absence of peptidoglycan contamination in the recombinant OmpA.

### B cell isolation and treatment

B cells were purified from spleen by negative selection (StemCell Technologies) according to the manufacturer's protocol. The purity of the cell preparations was determined by FACS analysis with phycoerythrin-conjugated anti-CD19 antibody. Routinely, the purity of the cell preparations was >95%. The cells were then washed in RPMI 1640 containing 2% FCS, 5 U/ml penicillin G, 5 µg/ml streptomycin, and 0.1% gentamycin. For inhibition studies, B cells were incubated either with TLR2 blocking antibody (purified monoclonal anti-mouse TLR2 antibody [Clone: T2.5]; InvivoGen), Mouse IgG1 isotype control, TLR4 blocking antibody (purified monoclonal antibody to mouse TLR4/MD2 [Clone: T2.5]; InvivoGen), Rat IgG2a isotype control, NF-κB nuclear translocation inhibitor (SN50 peptide; Santa Cruz Biotechnology Inc.), PTK inhibitor (Herbimycin A; Santa Cruz Biotechnology Inc.), p38 inhibitor (SB203580; Cell Signaling Technology), JNK inhibitor (SP600125; Cell Signaling Technology) or MEK1/2 inhibitor (U0126; Cell Signaling Technology) for 1 h prior to incubation with OmpA.

### Flow cytometry

B cells were cultured in presence of OmpA or media alone. Subsequently, cells were harvested and labeled with any one of FITC-conjugated anti-mouse CD80, CD86, MHC class II, TLR2 or PE-conjugated TLR4 (at 1:200 dilution) for 30 min on ice. Surface expression of TLR1 or TLR6 was detected by staining B cells with anti-mouse TLR1 or TLR6 purified antibody (at 1:200 dilution) followed by anti-rat IgG biotin (at 1:1000 dilution) and streptavidin PE (at 1:1500 dilution). The stained cells were examined on a FACSCalibur and results were analyzed using the CellQuest software (Becton Dickinson).

### RNA isolation and RT-PCR

Total RNA was extracted from B cells by RNAqueous- 4PCR kit (Ambion Inc.). The RNA was reverse transcribed using RETROscript kit (Ambion Inc.) and amplified by PCR with gene-specific primers for GAPDH, TLR1, TLR2, TLR4, and TLR6 using the specific murine primers. The primer sequences were as follows: GAPDH (forward: 5′-GAGTCTACTGGTGTCTTCACC-3′; reverse: 5′-TGTCATGGATGACCTTGGCCA-3′), TLR1 (forward: 5′-GACCAGGGCTGCTCT TATTTC-3′; reverse: 5′-CTAACAAACTCTGGGTCCAGG-3′), TLR2 (forward: 5′-C AAATCCTGGTTGACTGGCC-3′; reverse: 5′-TTCCTCTCAATGGGCTCCAG-3′), TLR4 (forward: 5′-TGGGAACAAACAGCCTGAGAC-3′; reverse: 5′-TCACACTG ACCACTGAACAC-3′), TLR6 (forward: 5′-AGCCTGAGGCATCTAGACCT-3′; reverse: 5′-GACTTCGTGCTGTCTCCGA-3′). The expression of housekeeping gene GAPDH was checked for each set of RT-PCR experiment.

### Cell proliferation and ELISPOT assay

For proliferation assay, purified B cells were labeled with 1 µM CFSE and stimulated with OmpA for 4 day. Cells were analyzed every 24 h by flow cytometry. To assess differentiation of B cells into ASCs, B cells were cultured for 1 h with or without the indicated inhibitors and then seeded into flat-bottom 96-well tissue culture plates. Cells were then cultured in presence of OmpA for 72 h, and then transferred to ELISPOT plates precoated with unlabeled anti-mouse Ig for 16–18 h at 37°C. The plates were washed, incubated with HRP-conjugated anti-IgM and anti-IgG Abs for 2 h at room temperature, and developed with AEC Chromogen (BD Biosciences). The plates were imaged and analyzed using an Immunospot plate reader.

### Cytokine ELISA

The quantities of IL-10, IL-6, IFN-γ, TNF-α, and IL-4 in culture supernatants were determined via sandwich ELISA (R&D Systems) following the manufacturer's instructions.

### Preparation of whole-cell, nuclear and cytoplasmic extracts and immunoblotting

B cells were incubated with OmpA for the indicated times. Whole-cell lysates were prepared by lysing cells in ice cold lysis buffer containing 20 mM Tris-HCl (pH-8.3), 150 mM NaCl, 1 mM EDTA, 1% Nonidet P-40, and protease and phosphatase inhibitors (5 mg/ml pepstatin A, 1 mM PMSF, 0.5 mM iodoacetamide, 1 mM sodium metavanadate, 10 mM sodium fluoride) for 30 min on ice.

Nuclear extracts were prepared as described by Barbeau et al., 1997 [25]. Briefly, 1×10^7^ cells, washed twice with cold PBS, were incubated for 15 min on ice in 400 µl of hypotonic buffer (buffer A: 10 mM HEPES [N-2-hydroxyethylpiperazine-N′-2-ethanesulfonic acid], pH-7.9; 10 mM KCl; 1.5 mM MgCl_2_; 1 mM dithiothreitol [DTT]; 0.5 mM phenylmethylsulfonyl fluoride; and protease inhibitor cocktail [1 µg/ml leupeptin, 1 µg/ml aprotinin, 10 µM pepstatin). Cells were lysed with 25 µl of Nonidet P-40 (10%). After brief vortexing and centrifugation, the supernatant (cytoplasm extract) was stored at -80°C until use while the pellet was resuspended with hypertonic buffer (buffer B: 20 mM HEPES, pH-7.9; 0.4 M NaCl; 1.5 mM MgCl_2_; 0.2 mM EDTA [ethylenediaminetetraacetic acid]; 1 mM DTT; 0.5 mM phenylmethylsulfonyl fluoride; 5% glycerol; and protease inhibitor cocktail [1 µg/ml leupeptin, 1 µg/ml aprotinin, 10 µM pepstatin) and gently agitated for 30 min at 4°C. After centrifugation, the supernatant (nuclear extract) was used immediately or stored at −80°C until used. The lysates were subjected to SDS-PAGE followed by electroblotted onto nitrocellulose membranes. Detection of Phospho-ERK, -p38, -JNK, ERK, p38, JNK, IκB, p65, α-Tubulin, Lamin B1 and β-Actin was conducted by immunostaining using their specific antibodies (at 1:1000 dilution) and horseradish peroxidase-conjugated (HRP) anti-IgG antibody (at 1:10,000 dilution). In order to examine global tyrosine phosphorylation, B cell lysates were probed with biotin-conjugated anti-phosphotyrosine antibody (at 1 µg/ml) followed by streptavidin-HRP antibody (at 1:4000 dilution). The protein bands were visualized by the enhanced chemiluminescence (ECL) assay (Amersham Pharmacia Biotech) following the manufacturer's instructions.

### Statistical analysis

The statistical significance of difference between the test groups was analyzed by Student's t-test (two-tailed) using SPSS 7.5 software. Results were expressed as the mean ± standard error of the mean (S.E.M.) where applicable, of three independent experiments and each experiment was performed in triplicate. Statistical significance was assumed at p<0.05.

## Results

### OmpA of *S. flexneri* 2a upregulates TLR2 mRNA and protein in B cells

B cells express multiple innate immune receptors and can be directly stimulated to produce antibodies or cytokines by microbial components containing Toll-like receptor agonists [24]. To ascertain the contribution of TLRs in recognition of OmpA, both TLRs mRNA and protein surface expression were measured in B cells. Cells were incubated with OmpA for 3 h and TLRs mRNA levels were examined by RT-PCR. OmpA induced expression of TLR2 and TLR6 mRNAs at 3 h compared to untreated cells (**Figure 1A**), whereas expression of TLR1 and TLR4 remained unchanged. GAPDH mRNA was used as a loading control. To determine whether regulation of TLR2 and TLR6 mRNAs were accompanied by there surface protein expression, flow cytometry analysis was performed, and representative histograms are shown in **Figure 1**. Incubation of B cells in presence of *S. flexneri* 2a OmpA for 6 h showed increased TLR2 (**Figure 1B**) and TLR6 surface expression (**Figure 1B**) with respect to untreated control, however expression of TLR1 and TLR4 remained unaltered (**Figure 1B**) following treatment with OmpA. Collectively, these results show that likely TLR2 in association with TLR6 contributing to the recognition and initiation of B cell response to OmpA.

**Figure 1:** OmpA of *S. flexneri* 2a induces expression of TLR2 and TLR6 in B cell. (**A**) Splenic B cells were stimulated with OmpA (5 µg/ml), total RNA was extracted after 3 h and subjected to RT-PCR using the appropriate primer. PCR products were quantified and expressed as the ratio of each product to GAPDH band density. The data are representative of three independent experiments. (**B**) Purified splenic B cells were incubated in the absence (red line) or presence (green line) of OmpA (5 µg/ml) for 6 h. Cells were harvested and assayed for cell surface expression of TLR1, TLR2, TLR4, and TLR6. The blue lines represent the isotype control antibodies. Representative data from three independent experiments are shown.

### OmpA stimulates phosphorylation of protein tyrosine kinases (PTKs) and MAP kinases as well as activates NF-κB downstream of TLR2

During B cell immune response the initial events involve rapid activation of numerous protein tyrosine kinases (PTK) that modulate various downstream signaling pathways including NF-κB and mitogen-activated protein (MAP) kinases result in an increase in the levels of transcription factors required for entering the cell cycle and differentiation pathways [26], [27]. To test this, we stimulated B cells with OmpA for different time intervals. Cell lysates were prepared and the profile of tyrosine-phosphorylated proteins was examined by immunoblotting. Compare to untreated cells, B cells cultured in presence of OmpA showed an increase in band intensity of many tyrosine-phosphorylated proteins (**Figure 2A**), representing a global increase in activation of proximal signaling molecules.

**Figure 2:** OmpA stimulates phosphorylation of protein tyrosine kinases, ERK, JNK and p38 and induces NF-κB activation. B cells were incubated with 5 µg/ml of OmpA for the indicated times, and cell lysates were probed for phosphotyrosine (pY) (**A**), and phosphorylated and total ERK, JNK and p38 (**B**). Representative blots from three independent experiments are shown. Arrows in the pY blot show bands with higher tyrosine phosphorylation. (**C**) B cells were purified from the spleen of BALB'/c mice, stimulated with OmpA (5 µg/ml) for the indicated times, and lysates were probed with phosphorylated and total IκBα. β-Actin was used as an internal control. The data is representative of three independent experiments. (**D**) B cells were cultured in absence and presence of OmpA for 30 min. The cytoplasmic (Cyto) and nuclear (Nuc) extracts were analyzed for p65, Lamin B1 (nuclear marker) and α-tubulin (Cytoplasmic marker) by Western blot analysis. The data shown are representative of three independent experiments.

To determine whether this higher magnitude of tyrosine phosphorylation influences downstream effector pathways, we examined the effect of OmpA on activation of MAP kinases, which include ERK, JNK and p38. OmpA induced phosphorylation of ERK, JNK and p38 in a time-dependent manner (**Figure 2B**). In addition, we determined the involvement of NF-κB in OmpA-induced signaling network. The translocation of NF-κB from cytoplasm to nucleus results from the phosphorylation and consequent degradation of IκB subunit from the NF-κB/IκB complex. The increased expression of p-IκB has been used as a measure of the activation of NF-κB [28]. To investigate if OmpA activates NF-κB in B cells, we monitored phosphorylation and degradation of IκBα by immunoblotting (**Figure 2C**). B cells treated with OmpA exhibited increased expression of p-IκB at 15 and 30 min time points (**Figure 2C**). To further confirm the involvement of NF-κB, we also examined nuclear translocation of NF-κB. OmpA induced nuclear translocation of p65 member of NF-κB family within 30 min of treatment (**Figure 2D**), demonstrating participation of NF-κB pathway in OmpA-mediated B cell immune response. Collectively, these data indicate that OmpA has the ability to activate proximal and distal B cell signaling molecules.

### OmpA increases surface expression of MHC II and CD86 on B cells

Since OmpA is a potent vaccine antigen and has the ability to activate adaptive immune response [9], we determined the expression of MHC II, CD80 and CD86 in response to OmpA on B cells. Purified B cells were incubated with OmpA for 24 h and expression of MHC II, CD80 and CD86 was measured by flow cytometric analysis. The histograms in **Figure 3** exhibit that OmpA was able to induce increased surface expression of MHC II and CD86, which were 2.5-fold (2.75±0.18, mean ± S.E., p<0.01) and 1.9-fold (2.15±0.19, mean ± S.E., p<0.01) more, respectively compared to untreated control, whereas the expression of CD80 (**Figure 3**) remained unaltered.

**Figure 3:** OmpA triggers expression of MHCII and CD86 on B cell. Splenic B cells were incubated without (red) or with (black) OmpA (5 µg/ml) for 24 h. Cells were harvested and assayed for cell surface expression of MHCII, CD80 and CD86. The shaded histograms indicate the isotype control antibodies. Representative data from three independent experiments are shown.

### OmpA induces B cell proliferation and differentiation into antibody secreting cells (ASCs)

Since our earlier study has been shown that immunization of mice with OmpA evokes strong induction of serum immunoglobulins [10], we therefore examined the direct effect of OmpA on B cell proliferation and differentiation *in vitro*. CFSE labeled splenic B cells were cultured in presence of OmpA for 96 h. OmpA treated B cells showed significantly enhanced CFSE dilution compared to untreated control in a dose-dependent manner (**Figure 4A**). In order to determine their differentiation into ASCs, B cells were stimulated with OmpA and the number of IgG- and IgM-secreting cells was quantified by ELISPOT. We found that OmpA stimulation induced a 4-fold increase in B cell differentiation into ASCs (**Figure 4B**). These results demonstrate that OmpA is a potent inducer of B cell activation.

**Figure 4:** OmpA evokes proliferation and differentiation of splenic B cells as well as induces secretion of IL-10 and IL-6. (**A**) CFSE-labeled B cells were cultured in medium alone or with an increasing concentration of OmpA for 96 h followed by flow cytometry. A representative of three independent experiments is shown and each experiment was done in triplicate. (**B**) The total number of ASCs (IgM + IgG-secreting cells) was analyzed by ELISPOT at the end of a 72 h culture period. Results are expressed as numbers of ASCs/10^5^ cells seeded and correspond to the mean ± S.E.M of quadruplicate determinations. **, p<0.01, relative to the untreated (media alone) group. (**C**) Purified splenic B cells were cultured in the absence or presence of indicated concentrations of OmpA for 72 h. The culture supernatants were assayed for IL-6 and IL-10 by enzyme-linked immunosorbent assay. The values are derived from IL-6 and IL-10 standard curves and represent the mean ± S.E.M of three independent experiments performed. **, p<0.01, relative to the untreated (media alone) group. (**D**) Time kinetics of IL-6 and IL-10 production by B cells incubated without or with OmpA (5 µg/ml). The values are derived from IL-6 and IL-10 standard curves and represent the mean ± S.E.M of three independent experiments performed. **, p<0.01, relative to the untreated (media alone) group.

### Induction of IL-10 and IL-6 by *S. flexneri* 2a OmpA in B cells

Besides producing antibodies, B cells can secrete numerous cytokines typically associated with innate or adaptive immune responses [15]. B cells were cultured in presence of increasing concentration of OmpA and the cell-free supernatants were assayed for the production of IL-6, IL-10, IFN-γ, TNF-α, and IL-4 by ELISA. OmpA stimulated IL-6 and IL-10 secretion in a dose- (**Figure 4C**) and time-dependent manner (**Figure 4D**). Production of IL-10 was induced at 48 h and elevated further at 72 h, whereas, IL-6 induced by OmpA peaked at 24 h and remained higher still 72 h (**Figure 4D**). However, OmpA did not evoke the secretion of IFN-γ, TNF-α, and IL-4 (data not shown). These data demonstrate that OmpA of *S. flexneri* 2a has the ability to induce secretion of both pro- and anti-inflammatory cytokines by B cells.

### OmpA-mediated-B cell differentiation and -cytokine production are TLR2 dependent

To confirm the prerequisite of TLR2 in OmpA-induced B cell effector functions, like antibody and cytokine production, an anti-TLR2 blocking antibody was employed. Blocking TLR2 significantly abrogated OmpA-induced differentiation of IgG ASCs (**Figure 5A**) compared to the results with OmpA alone or an isotype control antibody in the ELISPOT assay. Similarly, a dramatic reduction of cytokines, IL-6 and IL-10, of approximately 82% was observed by blocking TLR2 on B cell surface (**Figure 5B**). To further reinforce our understanding the role of TLR2 in the induction of B cell immune response, we also blocked TLR4 on the B cell surface using TLR4 mAb. OmpA was able to evoke B cell differentiation into antibody secreting cells (**Figure 5C**) as well as trigger secretion of cytokines (**Figure 5D**) even after blocking TLR4 on B cells, thus excluding the possibility of traces of LPS contamination in the recombinant OmpA and also confirms that the effect of OmpA on B cells is independent of TLR4. Collectively, these data provide evidences that *S. flexneri* 2a OmpA is recognized by TLR2 on B cell surface and subsequently activates downstream signaling cascades to modulate B cell effector functions, which are critical for the initiation of an adaptive immune response.

**Figure 5:** Involvement of TLR2 and protein tyrosine kinase in the OmpA-induced B cell differentiation and cytokine secretion. (**A, B**) B cells were incubated with anti-mouse TLR2 blocking antibody (100 ng/ml) or isotype (Mouse IgG1) control antibody (100 ng/ml) for 1 h at 37°C, followed by addition of OmpA (5 µg/ml) for a further 72 h. (**A**) The total number of ASCs (IgM + IgG-secreting cells) was analyzed by ELISPOT. Number of ASCs/10^5^ B cells. The results are the mean ± S.E.M of three independent experiments. ***, p<0.001, relative to OmpA treated group in the absence of TLR2 mAb. (**B**) The cell-free supernatants were assayed for IL-6 and IL-10 production by ELISA. The data are the mean ± S.E.M of three independent experiments. **, p<0.01, relative to OmpA treated group in the absence of TLR2 mAb. (**C, D**) B cells were incubated with anti-mouse TLR4/MD2 blocking antibody (100 ng/ml) or isotype (Rat IgG2a) control antibody (100 ng/ml) for 1 h at 37°C, followed by addition of OmpA (5 µg/ml) for a further 72 h. (**C**) The total number of ASCs (IgM + IgG-secreting cells) was analyzed by ELISPOT. Number of ASCs/10^5^ B cells. The results are the mean ± S.E.M of three independent experiments. (**D**) Production of IL-6 and IL-10 was examined by ELISA of the cell-free supernatants. The data represent the mean ± S.E.M of three independent experiments. (**E, F**) Purified B cells were cultured for 1 h with vehicle (DMSO) or the PTK inhibitor (Herbimycin A; 1 µM), followed by incubation with OmpA (5 µg/ml) for 72 h. (**E**) The total number of ASCs (IgM + IgG-secreting cells) was analyzed by ELISPOT. Number of ASCs/10^5^ B cells. The results are the mean ± S.E.M of three independent experiments. ***, p<0.001, relative to OmpA treated group in the absence of the inhibitor (DMSO). (**F**) Production of IL-6 and IL-10 was examined by ELISA in the cell-free supernatants. The data represent the mean ± S.E.M of three independent experiments. **, p<0.01, relative to OmpA treated group in the absence of the inhibitor.

### OmpA induces cytokine secretion and B cell differentiation through PTK activation

Protein tyrosine kinases play crucial role in cytokine production [29] and B cell proliferation [30] upon TLR ligation. Since our previous data had shown that OmpA triggers proximal protein tyrosine kinases (**Figure 2A**) and also stimulates B cell differentiation and cytokine secretion (**Figure 4**), here we determined whether PTK activity is required for these important B cell functions induced by *S. flexneri* 2a OmpA. Preincubation of B cells for 1 h with herbimycin A, a broad spectrum PTK inhibitor, absolutely diminished OmpA-induced B cell differentiation into ASCs (**Figure 5E**). Likewise, herbimycin also significantly reduced the OmpA-induced increase in the production of IL-6 and IL-10 by >80 (**Figure 5F**). These results demonstrate that OmpA-stimulated B cell differentiation and cytokine production are dependent on activation of PTKs.

### Involvement of NF-κB as well as ERK is essential for OmpA-stimulated cytokine secretion

The recognition of microbial components by TLRs effectively engages downstream signaling cascades such as, activation of NF-κB and mitogen-activated protein (MAP) kinases that culminate in the increased production of multiple cytokines, which are key players of the host immune response to bacterial infections [21]. Therefore, to gain further understanding into the mechanism of OmpA-induced production of cytokines, well-established inhibitors of NF-κB (SN50), p38 (SB203580), MEK1/2 (U0126) and JNK (SP600125) were employed. We first treated B cells with the inhibitors for 1 h before stimulating them with OmpA. After 72 h, ELISA was performed to detect production of IL-6 and IL-10 and the results exhibited that OmpA-stimulated production of cytokines was dependent on the NF-κB and ERK signaling as SN50 (**Figure 6A**) and U0126 (**Figure 6D**) compounds completely abolished the OmpA-dependent cytokine production. However, p38 (**Figure 6B**) and JNK inhibitors (**Figure 6C**) did not prevent the OmpA-induced upregulation of cytokines. These data indicate that both NF-κB and ERK pathways are critical for the cytokine production upon engagement of TLR2 by OmpA.

**Figure 6:** Effect of NF-κB-, p38-, JNK- and ERK-specific inhibitors on OmpA-stimulated production of IL-6 and IL-10. (**A-D**) B cells were purified from spleen, cultured for 1 h with vehicle or the inhibitors of NF-κB (SN50; 100 µg/ml), ***A***, p38 (SB203580; 5 µM), ***B***, JNK (SP600125; 5 µM), ***C***, MEK1/2 (U0126; 5 µM) ***D***, followed by incubation with OmpA (5 µg/ml). After 72 h of culture, the IL-6 and IL-10 levels in the cell supernatants were determined via sandwich ELISA. The data are the mean ± S.E.M of three independent experiments. **, p<0.01, relative to OmpA treated group in the absence of the inhibitor.

### OmpA-mediated B cell differentiation involves phosphorylation of ERK but not activation of MAP kinases or NF-κB

The extracellular signal-regulated kinase (ERK) plays central role in regulation of cell cycle progression, cell proliferation and differentiation of immune cells [31], [32]. In addition, NF-κB family members also control the transcription of genes that regulate cellular differentiation, survival and proliferation [33], [34], thereby regulate various aspects of innate and adaptive immune responses. Since our data showed that OmpA induces activation of both ERK and NF-κB as well as significantly enhances B cell differentiation into ASCs, we therefore examined whether activation of ERK or NF-κB is required in this process. Purified B cells were pretreated with the MEK1/2 inhibitor, U0126, or NF-κB inhibitor, SN50, for 1 h. Cells were then cultured in presence of OmpA and quantified the IgG- and IgM-secreting cells by ELISPOT. B cells pretreated with MEK1/2 inhibitor exhibited substantial reduction in the number of antigen specific ASCs with respect to cells stimulated OmpA alone (**Figure 7A**). Whereas, inhibition of NF-κB did not exert any effect on OmpA-induced B cell differentiation (**Figure 7B**).

**Figure 7:** Activation of ERK is critical for OmpA-induced differentiation of B cells into ASCs. B cells were purified from spleen, cultured for 1 h with vehicle or the inhibitors of MEK1/2 (U0126; 5 µM) ***A***, NF-κB (SN50; 100 µg/ml), ***B***, p38 (SB203580; 5 µM), ***C***, JNK (SP600125; 5 µM), ***D***, followed by incubation with OmpA (5 µg/ml) for 72 h. The total number of ASCs (IgM + IgG-secreting cells) was analyzed by ELISPOT. Number of ASCs/10^5^ B cells. The results are the mean ± S.E.M of three independent experiments. ***, p<0.001, relative to OmpA treated group in the absence of the inhibitor.

In order to further characterize the participation of additional signaling networks in OmpA-mediated B cell differentiation, B cells were pretreated with inhibitors, including p38 (SB203580) and JNK (SP600125), followed by incubation with OmpA for 72 h and the IgG- and IgM-secreting cells were enumerated by ELISPOT. As shown (**Figure 7** **, C and D**) the p38 and JNK inhibitors displayed no effect on OmpA-induced enhanced B cell differentiation. These observations confirm that ERK and not NF-κB, p38 or JNK is indispensible in the proliferation and differentiation of B cells induced by OmpA.

### TLR2 is critical in OmpA-induced nuclear translocation of NF-κB and ERK phosphorylation as well as antigen presentation

The observation that engagement of TLRs by microbial components mediates downstream signaling pathways that culminate in the activation of nuclear factor κB (NF-κB) and mitogen-activated protein (MAP) kinases, which results in the up-regulation of MHCII and costimulatory molecules [21], encouraged us to examine whether TLR2 is require for OmpA-induced activation of NF-κB and ERK as well as B cell antigen presentation. B cells isolated from spleen were incubated with mouse anti-TLR2 blocking antibody and then cultured with OmpA or medium alone. After 30 min, nuclear translocation of the p65 member of NF-κB family was determined. As shown in **Figure 8A**, OmpA was unable to stimulate nuclear translocation of p65 in TLR2 inhibited B cells, as compared with B cells cultured in presence of OmpA alone. To determine the role of TLR2 in OmpA-mediated phosphorylation of ERK, TLR2 inhibited B cells were cultured with OmpA for 5 min and our data revealed that blocking TLR2 almost completely abolished OmpA-mediated phosphorylation of ERK (**Figure 8B**). These data indicate that the TLR2 pathway is central in the effect of OmpA on activation of NF-κB and ERK in B cells. Importantly, we also analyzed the role of TLR2 in regulation of MHCII and CD86 expression on B cells in response to OmpA. B cells were incubated with TLR2 blocking antibody for 1 h followed by stimulation with OmpA for 24 h. The expression of MHCII and CD86 on B cells was analyzed by flow cytometry. OmpA-induced B cells upregulated the expression of MHCII (**Figure 8C**) and CD86 (**Figure 8D**), which were 3.2-fold (3.15±0.10, mean ± S.E., p<0.01) and 3.3-fold (3.25±0.12, mean ± S.E., p<0.01) higher, respectively compared to unstimulated cells. On the contrary, TLR2 blocking significantly prevented up-regulation of these molecules on B cells (**Figure 8, C and D**). These results indicate that recognition of OmpA via TLR2 on B cells is essential for the expression of MHCII and CD86, molecules known to be vital for antigen presentation to T cells, which is prerequisite for the development of an optimal T cell-dependent humoral immune response.

**Figure 8:** TLR2 is essential for OmpA-induced nuclear translocation of NF-κB, activation of ERK and expression of MHCII and CD86 on B cells. (**A**) B cells were incubated with anti-mouse TLR2 blocking antibody (100 ng/ml) for 1 h at 37°C prior to treatment with OmpA (5 µg/ml) for 30 min. The cytoplasmic (Cyto) and nuclear (Nuc) extracts were analyzed for p65, Lamin B1 (nuclear marker) and α-tubulin (Cytoplasmic marker) by Western blot analysis. The data shown are representative of three independent experiments. (**B**) B cells were pretreated with mouse anti-TLR2 blocking mAb (100 ng/ml) for 1 h. Cells were then stimulated with OmpA (5 µg/ml) for 5 min and cell lysates were probed for phosphorylated and total ERK. Representative blots from three independent experiments are shown. (**C, D**) B cells were incubated with anti-mouse TLR2 blocking antibody (100 ng/ml) for 1 h at 37°C (red line). Cells were then cultured in the absence (blue line) and presence (green line) of OmpA (5 µg/ml) for 24 h. Cells were harvested and assayed for cell surface expression of MHCII (**C**) and CD86 (**D**). The shaded histograms denote the isotype control antibodies. Representative data from three independent experiments are shown.

## Discussion

B cells play important role in antibacterial host defense through production of both antibodies and cytokines [12], [35]. In fact, antibodies are of the fundamental immune effectors induce by successful vaccines, since they bind specifically to pathogens to prevent the infections. We have previously reported that immunization of mice with OmpA evokes antigen specific IgG and IgA antibodies [10], suggesting an involvement of B-lymphocytes in OmpA-induced immune response. To explore the mechanism by which *S. flexneri* 2a OmpA activates B cells, we investigate the effect of OmpA on B cell signal transduction events allied with TLR2. In addition, we also identify the signaling pathways that bridge the innate activation of B cells via TLR2 with increased surface expression of MHCII and CD86, B cell proliferation and amplified B cell differentiation into ASCs, leading to the initiation of an adaptive immune response to OmpA.

B cells express a diverse array of innate immune receptors (TLRs) and can be directly stimulated to produce antibodies [23], [24], [36] or cytokines [15], [17] by the appropriate TLR ligands associated with pathogen upon encounter in the lymphatic system. Precisely, TLR2 and TLR4 can recognize a series of ligands, such as bacterial lipopeptides, LPS and other outer membrane bacterial components [37]. The initial TLR-mediated activation of B cells leads to the upregulation of co stimulatory CD80/CD86 and MHC-II receptors, thereby primes B cells for more abundant and efficient interactions with T cells and DCs [20], [38]. In fact Massari *et al*., [39] have demonstrated that B cell activation by the porin protein of *Neisseria meningitides* is dependent on TLR2 expression. Our data demonstrate that B cells express multiple TLRs, like TLR2, TLR4 and TLR6, but OmpA of *S. flexneri* 2a selectively induces increased expression of TLR2 and TLR6 as revealed by both flow cytometry and RT-PCR. These data indicate that TLR2 participates in recognition of OmpA by B cells. More interestingly, engagement of TLR2 by OmpA results in B cell activation, proliferation and differentiation into ASCs. To evaluate the significance of TLR2 in OmpA-mediated B cell immune response, TLR2 on B cell surface has been blocked using anti-TLR2 antibody. MHCII presentation of the processed antigen and expression of CD86 on B cells as well as B cell differentiation by OmpA of *S. flexneri* 2a have been dramatically reduced during TLR2 stalling, indicating that involvement of TLR2 is indispensible for the onset of B cell immune response to OmpA.

In addition to antibodies, B cells secrete various cytokines, including interleukin IL-1, IL-2, IL-4, IL-6, IL-10, IL-12, IFN-γ and TNF-α [17], classically modulate immune responses during bacterial infection. *S. flexneri* 2a OmpA induces release of IL-6 in both dose- and time-dependent manner. IL-6 is well known to enhance Ig secretion by activated B cells and causes their differentiation into plasma cells [40]. Mice deficient in IL-6 show reduced IgG2a production and have diminished mucosal IgA responses [41]. IL-6 plays crucial role in systemic immune defense against the bacterial pathogens, *Listeria monocytogenes* and *Citrobacter rodentium* [42], [43]. OmpA also increases secretion of IL-10 by B cells, which begin to release after 48 h of incubation and has been found to remain higher at 72 h. IL-10 is a potent anti-inflammatory cytokine, plays central role in regulating host immune responses to pathogens [44]. Deficiency of IL-10 can enhance inflammatory response to microbial challenge, leads to development of inflammatory bowel disease [45]. In response to *Shigella* invasion, it is well established that colonic epithelial cells produce a large array of pro-inflammatory cytokines and chemokines, such as IL-1β, IL-8 and IL-18, thereby trigger strong intestinal inflammation characteristic of shigellosis [46]. Hence, the OmpA-induced antibody and cytokine profile indicates that the protein has the ability to protect host in two levels, the increased differentiation of B cells into ASCs may lead to enhanced pathogen clearance and the amplified IL-10 release at later time point may limit unnecessary tissue disruptions caused by inflammation during *Shigella* infection [46].

B cell activation induced by OmpA has been evaluated by monitoring MHCII, CD80 and CD86 surface expression. In order to develop an effective adaptive immune response, T cells require two signals to become fully activated. Signal one is antigen (Ag) specific and is generated by binding of the T-cell receptor (TCR) to Ag-MHC complexes on the Ag-presenting cell (B cells, macrophages and dendritic cells). The second signal, a costimulatory signal, is generated by CD28 on the T cell interacting with CD80 (B7-1) or CD86 (B7-2) on an APC [47], [48]. Our data reveal that OmpA prompts high levels expression of MHCII and CD86 on B cells, suggesting that the increased MHCII and CD86 expression may serve to recruit more T cell help, thereby primes B cells for more abundant and efficient interactions with T cells. It is well known that T cell help to B cells promotes their affinity maturation, class-switch recombination and generation of memory [49], which are hallmarks of a potential vaccine antigen.

The molecular events occur following recognition of OmpA by TLR2 on B cell is not known. The activation of several protein tyrosine kinases (PTKs) plays the fundamental role in regulation of B cell development and effector functions [18], [50]. This initiates the formation of a ‘signalosome’ and signals emanate from the signalosome ultimately lead to the activation of multiple signaling cascades including NF-κB and MAP kinases [18], [50], [51]. Our data show that OmpA induces robust increase in phosphorylation of several tyrosine phosphorylated proteins and this overall increase in tyrosine phosphorylation also correlates with OmpA-mediated activation of downstream signaling molecules which involve NF-κB and ERK. Remarkably, we also show that pretreatment of B cells with herbimycin A decreases OmpA-mediated cytokine (IL-6 and IL-10) secretion and also blocks B cell differentiation into ASCs induced by OmpA, demonstrating a critical role of PTK in OmpA-induced B cell immune response downstream of TLR2 activation. These signal transduction pathways exactly mimic to those emerged following engagement of BCR by antigen or stimulation of CD40L. This data also corroborates with the findings of MacLeod *et al*., where they have shown that PorB of *Neisseria meningitides* acts via TLR2, triggers activation of tyrosine kinases and induces phosphorylation of ERK [30]. In an effort to confirm that the activation of NF-κB and ERK is dependent on recognition of OmpA by TLR2, TLR2 on B cell surface has been blocked using anti-TLR2 antibody. OmpA-induced nuclear translocation of NF-κB and phosphorylation of ERK have been greatly reduced following interference of TLR2. Collectively, our results suggest that OmpA recognition through TLR2 on B cells activates protein tyrosine kinases as well as downstream signaling molecules ERK and NF-κB, which, in turn, contribute to B cell differentiation into antibody secreting cells and cytokine production by B cells. NF-κB and ERK play critical role in cell cycle progression and cell proliferation in B cells [31], [32], [33]. Disruption of NF-κB activity exhibits defects in B cell development, activation and survival [34]. It has also been observed that conditional deletion of both ERK1 and ERK2 in germinal center B cells results in failure of plasma cell differentiation [52]. We therefore wanted to determine the role of NF-κB and ERK in OmpA-mediated release of cytokines by B cells and B cell differentiation into ASCs. Inhibition of NF-κB dramatically reduces OmpA-induced cytokine secretion, but B cell differentiation into ASCs remains unaffected, whereas, inhibition of ERK activation prevents both the cytokine release and differentiation of B cells. Taken together, these data demonstrate that there is divergence in requirement of signaling pathways in OmpA-induced B cell functions; NF-κB is pivotal for cytokine secretion, nonetheless both the cytokine production and B cell differentiation rely on ERK pathway.

Currently, we do not know the exact mechanisms of how recognition of OmpA by TLR2 promotes activation of non-receptor tyrosine kinases and distal signaling molecules like, NF-κB and ERK. One possibility is that engagement of TLR2 by OmpA results in the recruitment of Src family tyrosine kinases, such as Lyn, Fyn and Blk to the intracellular tail of TLR2 that contains a conserved region called the Toll/IL-1R homology (TIR) domain in association with MyD88, which in turn activates downstream signaling molecules, in particular NF-κB and ERK. Indeed, it has been found that Bruton's tyrosine kinase (Btk), a cytoplasmic non-receptor tyrosine kinase interacts with the intracellular TIR-domain in addition to other proteins within the multiprotein complex, like Mal, MyD88 and IRAK [54]. More interestingly, overexpression of a dominant negative mutant of Btk inhibits LPS-induced activation of NF-κB [53].

In conclusion, our study demonstrates that OmpA of *S. flexneri* 2a directly triggers and regulates B cell immune response, which is dependent on the interaction of OmpA with TLR2 on the cell surface. We also provide new insights on the potential mechanism of B cell response to OmpA. Once TLR2 on B cell surface recognizes OmpA, stimulates phosphorylation of multiple non-receptor tyrosine kinases, activates NF-κB and ERK and upregulates the surface expression of MHCII and CD86, which in turn modulates B cell proliferation and differentiation into antibody secreting cells as well as regulates production of cytokines (**Figure 9**) which are known to play crucial role in anti-bacterial host defense.

**Figure 9:** A hypothetical model for *S. flexneri* 2a OmpA-mediated activation of B cells and its role in regulation of host immune response.

Shigellosis represents a significant public health burden in developing countries, with about 160 million cases occurring annually, predominantly in children under the age of 5 years. Vaccination appears to be the effective and sustainable strategy to control shigellosis. The utmost complications to the use of vaccine against shigellosis in developing areas are the poor immune responses and lack of immunological memory. Studies have shown that TLR agonists namely CpG DNA, microbial lipoprotein, LPS, and flagellin can trigger activation of innate immune response [54]. Growing evidence also suggests the presence of TLR ligands in many established and experimental vaccines [55]. It has already been found that OmpA of *Klebsiella pneumoniae* binds to and activate macrophages and immature monocyte-derived dendritic cells (MDDC) in a TLR2-dependent manner [56]. In fact, *K. pneumoniae* OmpA has been identified as an excellent target for recombinant or conjugate subunit vaccine [56]. Furthermore, OmpA of *Escherichia coli* has been shown to stimulate dendritic cell activation and secretion of cytokines, critical to lift the immune response during infection [57]. Our study reveals that OmpA of *S. flexneri* 2a is a potent immunostimulatory TLR2 ligand. TLR2 engagement by OmpA is sufficient to induce B cell differentiation into antibody secreting cells and production of both pro- and anti-inflammatory cytokines. The present observations parallel previous study from our laboratory in which *S. flexneri* 2a OmpA had been demonstrated to evoke protective immune response in mice with induction of IgG and IgA antibodies in both the systemic and mucosal compartments [10] and perhaps contributing to identify a possible mechanism of OmpA-induced *in vivo* humoral immune response. The OmpA-induced increased expression of co-stimulatory CD86 and MHC-II receptors on B cells may be facilitating more efficient interactions with T cells, thereby enhancing the germinal center (GC) reaction and antibody affinity maturation that eventually giving rise to plasma and memory B cells, whose Ig genes encode antigen-specific, high-affinity and class-switched antibodies, leading to marked protective efficacy of OmpA *in vivo*. In this context it would be very interesting to examine whether *S. flexneri* 2a OmpA could retain long-term memory to protect the host from reinfection and should be evaluated in future studies. Furthermore, given the anti-inflammatory and antibody stimulating characteristics of IL-10, the delayed IL-10 production by B cells in response to OmpA may switch the inflammatory response observed in shigellosis [46] but at the same time possibly stimulate B cell proliferation and antibody secretion. Collectively, these findings indicate that OmpA of *S. flexneri* 2a modulate activation of B cells and humoral immune response through TLR2 and offer a novel visions towards the possible mechanism of protective immune response to virulent *Shigella* infection and further strengthen the implication of OmpA as a candidate vaccine antigen against shigellosis.

## Supporting Information

Figure S1 **Expression of recombinant his-tag OmpA.** Lane 1, Lonza ProSieve Color Protein molecular weight marker; lane 2, recombinant BL21 Star(DE3) *E. Coli* without IPTG; lane 3, recombinant BL21 Star(DE3) *E. Coli* with 0.25 mM IPTG; lane 4, Ni-NTA purified fraction; lane 5, Sephacryl S-200 HR purified fraction.
(TIF)

Figure S2 **OmpA of** ***S. flexneri*** **2a lacks NOD1 and NOD2 activities.** HEK 293 cells were transiently cotransfected with the pNFκB-MetLuc2-Repoter vector and the human NOD1 and NOD2 expression vectors, along with OmpA (5 µg/ml), M-triDAP or MDP for overnight. Relative luciferase activities in cell supernatants were analyzed by the Ready-To-Glow Secreted Luciferase Reporter Assay System. The data represent the mean ± S.E.M of three independent experiments. ***, p<0.001, relative to the untreated or OmpA treated group.
(TIF)

## References

[1] KotloffKL, WinickoffJP, IvanoffB, ClemensJD, SwerdlowDL, et al (1999) Global burden of *Shigella* infections: Implications for vaccine development and implementation of control strategies. Bull W H O 77: 651–666.10516787PMC2557719

[2] AshkenaziS, LevyI, KazaronovskiV, SamraZ (2003) Growing antimicrobial resistance of *Shigella* isolates. J Antimicrob Chemother 51: 427–429.1256271610.1093/jac/dkg080

[3] ChangA, KaurR, MichelLV, CaseyJR, PichicheroM (2011) *Haemophilus influenzae* vaccine candidate outer membrane protein P6 is not conserved in all strains. Human Vaccines 7(1): 102–105.2128553010.4161/hv.7.1.13351PMC3062244

[4] MesTH, Van PuttenJP (2007) Positively selected codons in immune-exposed loops of the vaccine candidate OMP-P1 of *Haemophilus influenzae* . J Mol Evol 64(4): 411–422.1747934210.1007/s00239-006-0021-2PMC1915622

[5] Vandeputte-RuttenL, BosMP, TommassenJ, GrosP (2003) Crystal structure of *Neisserial* surface protein A (NspA), a conserved outer membrane protein with vaccine potential. J Biol Chem 278(27): 24825–30.1271688110.1074/jbc.M302803200

[6] PoreD, ChowdhuryP, MahataN, PalA, YamasakiS, et al (2009) Purification and characterization of an immunogenic outer membrane protein of *Shigella flexneri* 2a. Vaccine 27: 5855–5864.1966058710.1016/j.vaccine.2009.07.054

[7] PoreD, ChakrabartiMK (2013) Outer membrane protein A (OmpA) from *Shigella flexneri* 2a: a promising subunit vaccine candidate. Vaccine 31: 3644–3650.2376453610.1016/j.vaccine.2013.05.100

[8] PoreD, MahataN, PalA, ChakrabartiMK (2010) 34-kDa MOMP of *Shigella flexneri* promotes TLR2-mediated macrophage activation with the engagement of NF-κB and p38 MAP kinase signaling. Mol Immunol 47: 1739–1746.2034748710.1016/j.molimm.2010.03.001

[9] PoreD, MahataN, ChakrabartiMK (2012) Outer membrane protein A (OmpA) of *Shigella flexneri* 2a links innate and adaptive immunity in a TLR2 dependent manner and with the involvement of IL-12 and nitric oxide (NO). J Biol Chem 287(15): 12589–601.2234363110.1074/jbc.M111.335554PMC3321007

[10] PoreD, MahataN, PalA, ChakrabartiMK (2011) Outer membrane protein A (OmpA) of *Shigella flexneri* 2a, induces protective immune response in a mouse model. PLoS ONE 6 e22663.2181836210.1371/journal.pone.0022663PMC3144247

[11] CasadevallA, PirofskiLA (2006) A reappraisal of humoral immunity based on mechanisms of antibody-mediated protection against intracellular pathogens. Adv Immunol 91: 1–44.1693853710.1016/S0065-2776(06)91001-3

[12] BebbingtonC, YarrantonG (2008) Antibodies for the treatment of bacterial infections: current experience and future prospects. Curr Opin Biotechnol 19: 613–619.1900076210.1016/j.copbio.2008.10.002

[13] BouazizJD, YanabaK, VenturiGM, WangY, TischRM, et al (2007) Therapeutic B cell depletion impairs adaptive and autoreactive CD4^+^ T cell activation in mice. Proc Natl Acad Sci U S A 104: 20882–20887.10.1073/pnas.0709205105PMC240923518093919

[14] ConstantS, SchweitzerN, WestJ, RanneyP, BottomlyK (1995) B lymphocytes can be competent antigen-presenting cells for priming CD4^+^ T cells to protein antigens in vivo. J Immunol 155: 3734–3741.7561077

[15] LundFE (2008) Cytokine-producing B lymphocytes-key regulators of immunity. Curr Opin Immunol 20: 332–338.1841733610.1016/j.coi.2008.03.003PMC2474694

[16] LintonPJ, BautistaB, BiedermanE, BradleyES, HarbertsonJ, et al (2003) Costimulation via OX40L expressed by B cells is sufficient to determine the extent of primary CD4 cell expansion and Th2 cytokine secretion in vivo. J Exp Med 197: 875–883.1266864710.1084/jem.20021290PMC2193894

[17] HarrisDP, HaynesL, SaylesPC, DusoDK, EatonSM, et al (2000) Reciprocal regulation of polarized cytokine production by effector B and T cells. Nat Immunol 1: 475–482.1110186810.1038/82717

[18] DeFrancoAL (1997) The complexity of signaling pathways activated by the BCR. Curr Opin Immunol 9: 296–308.920342110.1016/s0952-7915(97)80074-x

[19] PalmNW, MedzhitovR (2009) Pattern recognition receptors and control of adaptive immunity. Immunol Rev 227: 221–233.1912048710.1111/j.1600-065X.2008.00731.x

[20] PasareC, MedzhitovR (2005) Control of B-cell responses by Toll-like receptors. Nature 438: 364–368.1629231210.1038/nature04267

[21] KoppE, MedzhitovR (2003) Recognition of microbial infection by Toll-like receptors. Curr Opin Immunol 15: 396–401.1290027010.1016/s0952-7915(03)00080-3

[22] MedzhitovR, JanewayCAJ (1997) Innate immunity: the virtues of a nonclonal system of recognition. Cell 91: 295–298.936393710.1016/s0092-8674(00)80412-2

[23] PengSL (2005) Signaling in B cells via Toll-like receptors. Curr Opin Immunol 17: 230–236.1588611110.1016/j.coi.2005.03.003

[24] LanzavecchiaA, SallustoF (2007) Toll-like receptors and innate immunity in B-cell activation and antibody responses. Curr Opin Immunol 19: 268–274.1743387510.1016/j.coi.2007.04.002

[25] BarbeauB, BernierR, DumaisN, BriandG, OlivierM, et al (1997) Activation of HIV-1 long terminal repeat transcription and virus replication via NF-kappaB-dependent and -independent pathways by potent phosphotyrosine phosphatase inhibitors, the peroxovanadium compounds. J Biol Chem 272: 12968–12977.914890310.1074/jbc.272.20.12968

[26] NiiroH, ClarkEA (2002) Regulation of B-cell fate by antigen-receptor signals. Nat Rev Immunol 2: 945–956.1246156710.1038/nri955

[27] KurosakiT, HikidaM (2009) Tyrosine kinases and their substrates in B lymphocytes. Immunol Rev 228: 132–148.1929092510.1111/j.1600-065X.2008.00748.x

[28] HaydenMS, GhoshS (2004) Signaling to NF-κB. Genes Dev 18: 2195–2224.1537133410.1101/gad.1228704

[29] GengY, ZhangB, LotzM (1993) Protein tyrosine kinase activation is required for lipopolysaccharide induction of cytokines in human blood monocytes. J Immunol 151: 6692–6700.8258685

[30] MacLeodH, BhasinN, WetzlerLM (2008) Role of protein tyrosine Kinase and Erk1/2 activities in the toll-like receptor 2-induced cellular activation of murine B cells by *Neisserial* porin. Clin Vaccine Immunol 15: 630–637.1828758010.1128/CVI.00435-07PMC2292646

[31] ChangL, KarinM (2001) Mammalian MAP kinase signaling cascades. Nature 410: 37–40.1124203410.1038/35065000

[32] ChambardJC, LeflochR, PouysségurJ, LenormandP (2007) ERK implication in cell cycle regulation. Biochim Biophys Acta 1773: 1299–1310.1718837410.1016/j.bbamcr.2006.11.010

[33] GerondakisS, SiebenlistU (2010) Roles of the NF-κB pathway in lymphocyte development and function. Cold Spring Harb Perspect Biol 2: a000182.2045295210.1101/cshperspect.a000182PMC2857169

[34] LiouHC, ShaWC, ScottML, BaltimoreD (1994) Sequential induction of NF-kappa B/Rel family proteins during B-cell terminal differentiation. Mol Cell Biol 14: 5349–5359.803581310.1128/mcb.14.8.5349-5359.1994PMC359054

[35] PistoiaV (1997) Production of cytokines by human B cells in health and disease. Immunol Today 18: 343–350.923883810.1016/s0167-5699(97)01080-3

[36] GerondakisS, GrumontRJ, BanerjeeA (2007) Regulating B-cell activation and survival in response to TLR signals. Immunol Cell Biol 85: 471–475.1763769710.1038/sj.icb.7100097

[37] TakedaK, KaishoT, AkiraS (2003) Toll-like receptors. Annu Rev Immunol 21: 335–376.1252438610.1146/annurev.immunol.21.120601.141126

[38] Meyer-BahlburgA, RawlingsDJ (2008) B cell autonomous TLR signaling and autoimmunity. Autoimmun Rev 7: 313–316.1829573610.1016/j.autrev.2007.11.027PMC2763483

[39] MassariP, HennekeP, HoY, LatzE, GolenbockDT, et al (2002) Cutting edge: Immune stimulation by *Neisserial* porins is toll-like receptor 2 and MyD88 dependent. J Immunol 168: 1533–1537.1182347710.4049/jimmunol.168.4.1533

[40] MuraguchiA, HiranoT, TangB, MatsudaT, HoriiY, et al (1988) The essential role of B cell stimulatory factor 2 (BSF-2/IL-6) for the terminal differentiation of B cells. J Exp Med 167: 332–344.325800610.1084/jem.167.2.332PMC2188837

[41] KopfM, BaumannH, FreerG, FreudenbergM, LamersM, et al (1994) Impaired immune and acute-phase responses in interleukin-6-deficient mice. Nature 368: 339–342.812736810.1038/368339a0

[42] DalrympleSA, LucianLA, SlatteryR, McNeilT, AudDM, et al (1995) Interleukin-6-deficient mice are highly susceptible to Listeria monocytogenes infection: correlation with inefficient neutrophilia. Infect Immun 63: 2262–2268.776860710.1128/iai.63.6.2262-2268.1995PMC173295

[43] DannSM, SpehlmannME, HammondDC, IimuraM, HaseK, et al (2008) IL-6-dependent mucosal protection prevents establishment of a microbial niche for attaching/effacing lesion-forming enteric bacterial pathogens. J Immunol 108: 6816–26.10.4049/jimmunol.180.10.6816PMC269606318453602

[44] MosserDM, ZhangX (2008) Interleukin-10: new perspectives on an old cytokine. Immunol Rev 226: 205–18.1916142610.1111/j.1600-065X.2008.00706.xPMC2724982

[45] O'GarraA, BarratFJ, CastroAG, VicariA, HawrylowiczC (2008) Strategies for use of IL-10 or its antagonists in human disease. Immunol Rev 223: 114–31.1861383210.1111/j.1600-065X.2008.00635.x

[46] SchroederGN, HilbiH (2008) Molecular Pathogenesis of *Shigella* spp.: controlling host cell signaling, invasion, and death by type III secretion. Clin Microbiol Rev 21: 134–156.1820244010.1128/CMR.00032-07PMC2223840

[47] GreenfieldEA, NguyenKA, KuchrooVK (1998) CD28/B7 costimulation: a review. Crit Rev Immunol 18: 389–418.978496710.1615/critrevimmunol.v18.i5.10

[48] Marshall-ClarkeS, TaskerL, HeatonM, ParkhouseR (2003) A differential requirement for phosphoinositide 3-kinase reveals two pathways for inducible upregulation of major histocompatibility complex class II molecules and CD86 expression by murine B lymphocytes. Immunology 109: 102–108.1270902310.1046/j.1365-2567.2003.01638.xPMC1782951

[49] XuZ, ZanH, PoneEJ, MaiT, CasaliP (2012) Immunoglobulin class-switch DNA recombination: induction, targeting and beyond. Nat Rev Immunol 12: 517–531.2272852810.1038/nri3216PMC3545482

[50] KurosakiT, HikidaM (2009) Tyrosine kinases and their substrates in B lymphocytes. Immunol Rev 228: 132–148.1929092510.1111/j.1600-065X.2008.00748.x

[51] NiiroH, ClarkEA (2002) Regulation of B-cell fate by antigen-receptor signals. Nat Rev Immunol 2: 945–956.1246156710.1038/nri955

[52] YasudaT, KometaniK, TakahashiN, ImaiY, AibaY, et al (2011) ERKs induce expression of the transcriptional repressor Blimp-1 and subsequent plasma cell differentiation. Sci Signal 4: ra25.2150518710.1126/scisignal.2001592

[53] JefferiesCA, DoyleS, BrunnerC, DunneA, BrintE, et al (2003) Bruton's tyrosine kinase is a Toll/interleukin-1 receptor domain-binding protein that participates in nuclear factor kappaB activation by Toll-like receptor 4. J Biol Chem 278: 26258–26264.1272432210.1074/jbc.M301484200

[54] BartonGM, MedzhitovR (2003) Toll-like receptor signaling pathways. Science 300: 1524–1525.1279197610.1126/science.1085536

[55] LahiriA, DasP, ChakravorttyD (2008) Engagement of TLR signaling as adjuvant:towards smarter vaccine and beyond. Vaccine 26: 6777–6783.1883557610.1016/j.vaccine.2008.09.045

[56] Pascale JeanninP, MagistrelliG, GoetschL, HaeuwJF, ThieblemontN, et al (2002) Outer membrane protein A (OmpA): a new pathogen-associated molecular pattern that interacts with antigen presenting cells-impact on vaccine strategies. Vaccine 20: A23–A27.1247742410.1016/s0264-410x(02)00383-3

[57] TorresAG, LiY, TuttCB, XinL, Eaves-PylesT, et al (2006) Outer membrane protein A of *Escherichia coli* O157:H7 stimulates dendritic cell activation. Infect Immun 74: 2676–2685.1662220410.1128/IAI.74.5.2676-2685.2006PMC1459721

